# Rare Overlap of Granulomatosis With Polyangiitis in a Patient With Rheumatoid Arthritis

**DOI:** 10.7759/cureus.19303

**Published:** 2021-11-06

**Authors:** David Grzybacz, Ndausung Udongwo, Remi Ashkar, Amanda Woodford, Sobaan Taj, Mohammad A Hossain, James Cosentino

**Affiliations:** 1 Internal Medicine, Jersey Shore University Medical Center, Neptune City, USA; 2 Medicine, Hackensack Meridian School of Medicine, Nutley, USA; 3 Pulmonology, Jersey Shore University Medical Center, Neptune City, USA

**Keywords:** lung biopsy, cavitary lesions, anca-associated vasculitis, rheumatoid arthritis (ra), granulomatosis with polyangiitis (gpa)

## Abstract

Granulomatosis with polyangiitis (GPA) is a systemic small/medium-sized vessel vasculitis, which is a member of the family of antineutrophil cytoplasmic auto-antibody-associated vasculitides. This disorder affects multiple organs as it is a systemic disease, but overlapping with rheumatoid arthritis is extremely rare, with few cases reported in the medical literature. We report a case of a 55-year-old female with a history of rheumatoid arthritis who presented with recurrent upper/lower respiratory tract symptoms that responded poorly to antibiotics. The patient had elevated antiproteinase antibodies, ANCA IgG titer with a cytoplasmic staining pattern, proteinuria, hematuria, chest imaging showing cavitating and non-cavitating masses, and biopsies of lung and nasal tissue confirming the diagnosis of GPA. Our patient was given immunosuppressant therapy and improvement in lab work and clinical symptoms were seen throughout the course of treatment. This case report is unique as GPA usually rarely presents with rheumatoid arthritis (RA), but in this case, the patient had a history of rheumatoid arthritis with a new biopsy-proven GPA. This case report will help future physicians to better diagnose similar cases and help to facilitate clinical recognition and treatment for the same.

## Introduction

Granulomatosis with polyangiitis (GPA) is one of the few small/medium-sized vessel vasculitides with a wide systemic distribution [1]. It is an antineutrophil cytoplasmic antibody (ANCA)-associated granulomatous inflammatory process that has a predilection for the upper and lower respiratory tracts and the kidneys. GPA has variable clinical presentations, which may cause a delay in diagnosis and prompt management. It has a mortality rate of about 80% if left untreated [1,2]. A detailed history, imaging findings, and biopsy results could help in early treatment, which may reduce mortality. We present a case of a 55-year old female with a history of rheumatoid arthritis (RA) who presented with recurrent upper/lower respiratory tract symptoms and responded poorly to antibiotics. Biopsy-proven GPA led to appropriate management with the resolution of symptoms. Although other overlap syndromes have been described in association with rheumatoid arthritis, ANCA-associated vasculitides overlapping with RA is extremely rare, with few cases described in the medical literature [3]. Furthermore, an overlap between RA and cytoplasmic-ANCA (c-ANCA)-associated GPA is rare, and there should be high suspicion for GPA in patients with similar symptoms who were previously diagnosed with RA.

## Case presentation

A 55-year- old female with a past medical history of RA, diagnosed five years ago with a positive rheumatoid factor of 118 IU/mL (normal reference < 14 IU/mL), presented to the emergency department (ED) with complaints of worsening sinus congestion that started three months prior to admission. Symptoms included post-nasal drip, worsening cough, night sweats, perforated nasal septum, episodes of nosebleeds, and a 15-pound unintentional weight loss during this period. She had also recently noticed a collapse of the bridge of her nose. Of note, she had multiple visits to otolaryngologists for the same complaints. Antibiotics and bi-nasal washes did not provide any relief from her symptoms. She denied any chest pain, fever, chills, loss of smell/taste, shortness of breath, nausea, vomiting, or recent sick contacts. Home medications were methotrexate, hydroxychloroquine, folic acid, and ibuprofen. Family history was remarkable for breast cancer in the mother and melanoma in the brother. She denied any tobacco or recreational drug use in the past and drank alcohol occasionally. 

Her initial vital signs showed a blood pressure of 132/60 mmHg, heart rate of 102 beats per minute, respiratory rate of 20 breaths per minute, temperature of 97℉, and oxygen saturation of 97% on room air. Examination of the patient’s nose showed saddle nose deformity with septal perforation. The cardiopulmonary examination was remarkable for tachycardia and diffuse lung crackles bilaterally on auscultation. The musculoskeletal examination was significant for mild swelling of the left third metacarpophalangeal (MCP) joint, mild fullness of the left third MCP joint with mild tenderness, and mild tenderness of the second and third proximal interphalangeal (PIP) joints. Initial laboratory analysis is shown in Table 1. 

**Table 1:** Laboratory results c-ANCA: cytoplasmic antineutrophil cytoplasmic antibody; ANCA: antineutrophil cytoplasmic antibody; RBCs: red blood cells; HPF: high power field

Name of the test	Results	Reference range
Hemoglobin (g/dL)	8.8 (g/dL)	12.0-16.0 (g/dL)
White blood cells (10^3^/uL)	12.9 (10^3^/uL)	4.5-11.0 (10^3^/uL)
Sodium (mmol/L)	137 (mmol/L)	136-145 (mmol/L)
Potassium (mmol/L)	3.5 (mmol/L)	3.5-5.0 (mmol/L)
Blood urea nitrogen (BUN) (mg/dL)	10 (mg/dL)	5-25 (mg/dL)
Creatinine (mg/dL)	0.65 (mg/dL)	0.44-1.0 (mg/dL)
Antiproteinase-3 antibodies (U/mL)	10.4 (U/mL)	0.0-3.5 (U/mL)
Cytoplasmic antineutrophil cytoplasmic antibody (c-ANCA) IgG titer	1:40	<1:20
Perinuclear ANCA	<1:20	<1:20
Anti-myeloperoxidase antibodies	<9.0 (U/mL)	0-9.0 (U/mL)
Anti-glomerular basement membrane antibodies (units)	2 (units)	0-20 (units)
Urinalysis; red blood cells/high power field (RBCs/HPF)	3-10	0-2
Urine protein/creatinine ratio	269 (mg/g)	0-200 (mg/g)

Initial chest x-ray revealed multiple cavitating and non-cavitating masses scattered throughout the lungs bilaterally, largest on the right, measuring 7.4 cm in diameter (Figure 1).

**Figure 1:** Chest x-ray showing multiple bilateral non-cavitating and cavitating masses (red arrows)

Computed tomography angiography of the chest revealed cavitary and non-cavitary masses with the largest cavitary lesion in the superior segment of the right lower lobe (Figures 2A, 2B). 

**Figure 2:** Computed tomography angiography of the chest showing non-cavitary lesions (A: lower red arrow) and cavitary lesions (A: upper red arrow and B: both red arrows), with the largest cavitary lesion being seen in the superior segment of the right lower lobe (B: lower red arrow)

Lung biopsy of tissue from the right lower lobe showed lung parenchyma with organizing fibrosis, marked histiocytic response with focal areas forming vague granulomas with fibrinoid necrosis, acute and chronic inflammation, and single vessel with vasculitis (best appreciated on elastin stain) (Figures 3A-3D). A biopsy of left nasal tissue revealed respiratory mucosa demonstrating necrotizing granulomatous inflammation associated with polarizable foreign material and a focus of small vessel vasculitis. A kidney biopsy was not performed. 

**Figure 3:** Lung biopsy of tissue from the right lower lobe shows lung parenchyma with organizing fibrosis (A and C), marked histiocytic response with focal areas forming vague granulomas with fibrinoid necrosis (D), acute and chronic inflammation, and single vessel with vasculitis best appreciated on elastin stain (B)

Given the patient’s confirmed GPA, the patient was initially started on a rituximab-based induction regimen of 375 mg/m^2^ per week for four weeks along with a prednisone taper with an initial dose of 60 mg daily and subsequent taper down to 5 mg daily. Three months after initiation of treatment, antiproteinase-3 antibodies continued to be elevated at 7.2 U/mL but c-ANCA was normal at <1:20. Chest x-ray three months after initiation of treatment continued to show bilateral cavitary pulmonary parenchymal abnormalities but associated wall thickening was significantly diminished (Figure 4). Notably, the patient’s urine protein/creatinine ratio increased from 269 mg/g to 444 mg/g and her urinalysis revealed 11-30 RBCs/HPF, increased from 3-10 RBCs/HPF three months prior. The patient’s creatinine was also increased from 0.5-0.7 mg/dL on initial presentation to >1.1 mg/dL. Because of concern for new-onset renal involvement in the setting of confirmed GPA, the patient was transitioned to oral cyclophosphamide as there was concern that rituximab was not leading to clinical remission. She was initially started on a 2 mg/kg dose of cyclophosphamide with up-titration to 3 mg/kg after one month, but the dose was titrated back down to 2 mg/kg one month later given elevated transaminases. After approximately three months of cyclophosphamide, the patient’s dose was reduced to 1 mg/kg after sustained clinical improvement, as evidenced by laboratory analysis, imaging studies, and clinical signs and symptoms. 

**Figure 4:** Chest x-ray done three months after initial treatment of GPA The image shows improvement in cavitary lesions when compared with prior imaging as seen in Figure 1. GPA: granulomatosis with polyangiitis

Six months after initiation of treatment, antiproteinase-3 antibodies normalized at <3.5 U/mL, and c-ANCA continued to be normal at <1:20. Repeat CT chest without contrast revealed resolution of the previously noted cavitary mass lesions. Notably, the patient’s urine protein/creatinine ratio improved to normal (<200 mg/g). The patient’s urinalysis also improved, showing only 3-10 RBCs/HPF compared to 11-30 RBCs/HPF 3 months prior. The patient’s creatinine was also stable at around 1.1 mg/dL. After nine months of treatment, the patient was transitioned off of cyclophosphamide and started maintenance therapy with rituximab.

## Discussion

An overlap syndrome of GPA in association with RA appears to be relatively rare, with less than 20 articles found during the literature review [4]. In our patient with established RA, it was important to consider GPA in the differential diagnosis given the patient’s recurrent upper/lower respiratory tract symptoms, septal nose deformity, imaging results, and laboratory abnormalities with ultimate confirmation of the diagnosis with biopsies of nasal and lung tissues. ANCA-associated vasculitis, in general, is made up of three distinct clinical conditions: granulomatosis with polyangiitis (GPA), microscopic polyangiitis (MPA), and eosinophilic granulomatosis with polyangiitis (EGPA) [5]. Most often, these conditions are characterized by ANCA that is reactive against one of two antigens, proteinase-3 or myeloperoxidase. Antiproteinase-3 antibodies are a subgroup of antineutrophil cytoplasmic antibodies found most often in patients with active Wegener’s granulomatosis, but in a study of 32 patients with rheumatoid arthritis, anti-proteinase 3 antibodies were not detected [5]. For our patient, her initial antiproteinase-3 antibody level was elevated at 10.4 U/mL, which is consistent with active GPA. Notably, antibodies against myeloperoxidase were not evident in the laboratory evaluation of our patient. Previous research has shown that the presence of antibodies to proteinase-3 is most often associated with GPA while antibodies to myeloperoxidase are most often associated with the other two ANCA-associated vasculitides (EGPA and MPA) [4,6]. Additionally, a c-ANCA staining pattern is most often associated with GPA as c-ANCA antibody is against neutrophil proteinase 3, while a perinuclear antineutrophil cytoplasmic antibody (p-ANCA) staining pattern is associated with EGPA and MPA as the p-ANCA antibody is against neutrophil myeloperoxidase [7].

Regarding treatment, several different strategies are used clinically to treat patients with GPA with two distinct phases, induction and maintenance [8]. The overall approach to treatment differs based on whether or not there is the presence of organ- or life-threatening disease. For this patient, given the presence of significant pulmonary involvement, her treatment was based on guidelines for organ-threatening disease. In such patients, induction therapy usually involves the use of either rituximab or cyclophosphamide with glucocorticoids, while maintenance therapy is often initiated with rituximab after successful remission with immunosuppressive therapy [8]. An interesting aspect of this case was that despite therapy with rituximab and improvement in the patient’s pulmonary manifestations and laboratory findings while receiving this treatment, the patient’s renal function worsened as evidenced by increased serum creatinine, increased urinary protein/creatinine ratio, and increased RBCs/HPF on urinalysis, therefore raising concern for new-onset renal involvement, a common manifestation of GPA. Because of these concerns, the patient was transitioned from rituximab to cyclophosphamide, another drug commonly used in the treatment of GPA, while also continuing on glucocorticoids. Notably, after further induction treatment with cyclophosphamide, the patient experienced sustained clinical improvement noted on imaging, laboratory results, and clinical signs and symptoms. Notably, the patient’s urine protein/creatinine ratio improved to normal (<200 mg/g), the patient’s urinalysis showed only 3-10 RBCs/HPF compared to 11-30 RBCs/HPF three months prior, and the patient’s creatinine was also stable at around 1.1 mg/dL. After nine months of treatment, the patient was transitioned off of cyclophosphamide and started maintenance therapy with rituximab. Overall, clinicians often try to limit the use of cyclophosphamide over a long-term period given its known risks of toxicity [9]. However, given our patient’s new renal findings, it was determined that cyclophosphamide was a prudent option for immunosuppressive therapy, albeit until remission was achieved. The patient will continue with maintenance therapy for at least three years in line with clinical guidelines given her multiple risk factors for relapse, including PR3-ANCA seropositivity and pulmonary involvement [10]. Through confirming the diagnosis of GPA in a patient with previously diagnosed RA, the patient was started on appropriate therapeutic management with subsequent clinical resolution of her presenting symptoms, imaging findings, and laboratory abnormalities. 

## Conclusions

Granulomatosis with polyangiitis associated with RA is a rare form of ANCA-associated vasculitis autoimmune overlap syndrome. Prompt recognition in patients with similar clinical scenarios could facilitate early diagnosis with appropriate management, which may help reduce mortality. There should be a high index of suspicion for this overlap syndrome (RA/GPA overlap) in patients with a prior history of RA just like our patient.
